RETRACTED

# Study on the Correlation between Morphology and Distribution of Common Psoriasis Lesions

**DOI:** 10.1155/2022/6963630

**Published:** 2022-03-23

**Authors:** Qiang Li, Yuanwen Jiang

**Affiliations:** ^1^Department of Dermatology, Air Force Medical Center, PLA, Beijing 100142, China; ^2^Dermatology Department, Affiliated Hospital of Youjiang Medical University for Nationalities, Baise, Guangxi 533000, China

## Abstract

**Objective:**

Through the analysis of the morphological distribution of psoriasis lesions, we can study the relationship between psoriasis lesions and age, gender, and course of disease and dialectically look at the location of lesion morphology and the impact of course of disease on it, so as to provide more basis for the treatment of psoriasis.

**Method:**

Through a questionnaire survey of 512 patients in the dermatology clinic of a well-known traditional Chinese medicine hospital in Jiangsu Province, their symptoms met the diagnostic criteria of psoriasis in Chinese clinical dermatology. The current situation of psoriasis was analyzed by literature analysis, and the collected data were analyzed by general mean analysis, analysis of variance, and descriptive analysis.

**Result:**

There were some differences in the proportion of male to female in 512 patients. It is possible to conclude that male incidence rate is higher than that of women. It can be deduced from bad habits such as heavy drinking and smoking in male life. Bad habits can reduce male immunity and cause disease. The distribution of skin lesions in different parts shows that the skin is more affected by the outside world, which leads to the repeated attack of psoriasis. The incidence of chest, scalp, and upper arm is also relatively high. There have been similar demonstrations in relevant medical data, which may be related to the vascular density in them. Some substances that induce psoriasis in the dense blood vessels are easy to accumulate here, leading to the pathogenic bacteria to induce the onset of psoriasis.

**Conclusion:**

By studying the distribution of psoriasis lesions and the correlation between lesions, gender, and disease course, we can improve the dialectical treatment of psoriasis, which has reference significance, and provide a new thinking direction for the treatment system theory of psoriasis.

## 1. Introduction

Psoriasis is a common autoimmune disease, which is stubborn and easy to relapse. Routine treatment can not achieve the effect of radical cure. The common symptoms of clinical manifestations are erythema and scales. Symptoms can be seen all over the body, mostly in young and strong years. The disease rate of men is greater than that of women. It usually occurs on the scalp and limbs, especially in winter.

RETRACTED

There are many kinds of skin lesions in general psoriasis. The small can be the size of a needle, and the large can extend to the whole body. The number and shape are different. Pathologically, the etiology of psoriasis is mainly related to heredity, autoimmune system, endocrine system, mental factors, and emotions.

According to Yuying and Dongmei [1], a Western doctor, believes that psoriasis is a chronic disease with problems in the immune system, and the cause of the disease has not yet been identified. At present, it is considered that psoriasis is related to family heredity and lack of immune function, as well as to microorganisms. This paper focuses on the microecological imbalance of skin and mucosa. It is considered that the imbalance of microbial ecological environment is very likely to induce excessive immune response of susceptible hosts and lead to continuous inflammation of autoimmune system. According to Wang et al. [2], there are about 6.5 million patients with psoriasis in China, and this number is still growing, but there is a lack of relevant data to study psoriasis. In this paper, the medical history of more than 6000 patients was analyzed, and their onset characteristics and clinical symptoms were helpful to understand the symptoms of psoriasis, so as to optimize the treatment plan and patient follow-up management in the future.

Psoriasis is a chronic skin disease that can be involved in the whole body cortex, and the shape of skin lesions is diverse, the location of onset is uncertain, and environmental and genetic factors are related to the onset, so it can not be targeted treatment. Western medicine generally adopts immune administration. This treatment is characterized by continuous administration according to the severity of the disease, but it is not recommended to use large doses for a long time, and relapse after stopping the drug. In recent years, the emergence of biological agents has reduced a lot of pain to patients, but it is still unable to achieve a radical cure.

According to Xinyu et al. [3], the pathology of psoriasis changes the morphology of the surface layer of the skin, mainly manifested in lymphocyte-based inflammatory diseases such as hyperkeratosis, surface thickening, vasodilation, and congestion. At present, the combination of Chinese and Western medicine is mainly used, including glucocorticoids and traditional Chinese medicine compound granules, which can only alleviate the disease to a certain extent and can not achieve the curative effect. The bioscience proposed in this paper is biological agents, and its action mechanism is only to alleviate the symptoms and can not achieve a radical cure.

RETRACTED

Most of the drugs used for psoriasis are given routine treatment in general specialized hospitals. The scheme of combining Chinese and Western medicine is adopted. Western medicine is commonly used in glucocorticoids, which has obvious effect, but it is not suitable for long-term and continuous large-scale use. Pay attention to side effects. According to the clinical manifestations, TCM carries out syndrome differentiation and treatment. The treatment of blood heat type is based on clearing heat, cooling blood, and promoting blood circulation, and the treatment of blood dryness type is based on nourishing blood and moistening skin, promoting blood circulation, and dispersing wind. However, the course of psoriasis is long-lasting and easy to relapse. Overtreatment will cause adverse reactions and health discomfort. The purpose of this study is to explore the distribution of lesion morphology in different stages of psoriasis and whether the distribution of lesion morphology is related to gender and course of psoriasis.

## 2. Data and Methods

### 2.1. Research Object

The subjects selected in this study were outpatients from the dermatology department of a well-known traditional Chinese medicine hospital in Jiangsu Province. The patients were treated from January 2020 to June 2020. There are a total of 512 patients with psoriasis vulgaris in varying degrees, including 283 males and 229 females, aged 2-81 years, with an average age of 31.5 ± 4.3 years. The shortest medical history was two months, and the longest was 48 years. There were 186 cases in the onset stage, including 105 males and 81 females, 227 cases in the stable stage, including 122 males and 105 females, and 99 cases in the recovery stage, including 56 males and 43 females. The symptoms of all patients met the diagnostic criteria of routine psoriasis.

In Figure 1, although the pathological incidence rate of psoriasis is higher than that of women, there is no scientific basis for demonstrating the reason why men are higher than women. Based on the different living habits of men and women, male patients smoke more and drink a lot. Clinically, these may be the reasons for the high incidence of male patients in women.

#### 2.1.1. Diagnostic Criteria of Western Medicine

The relevant pathological indexes and skin microbiological test results were tested by blood sampling. Refer to Chinese clinical dermatology for details. The rash is mainly characterized by the formation of red papules or macular papules on the skin surface, with obvious boundary layers, which can expand or appear in a large area with the development of the disease. There will be dandruff on the surface. After scratching, the fish scale dandruff will disappear, and there will be a smooth membrane, covered with small bleeding points below. These manifestations are also the basic characteristics of the diagnosis of psoriasis. The rash forms are drop-like, coin-like, irregular map-like, and mixed. Ring and band-like are rare. In addition, there are different shell-like rash forms, but generally speaking, its boundary is clear. The skin lesions can occur all over the body. It can be seen in the skin that the scalp hair is twisted in a bundle, and it can be seen in the nails. Qualitative changes can be seen in the nails, accompanied by itching, greatly affecting the quality of life.

RETRACTED

#### 2.1.2. Patient Case Collection Scheme

Select the clinical patients who meet the diagnostic criteria of psoriasis vulgaris by Western medicine, have clear consciousness, and can cooperate with the investigation, and the patients have the right to know and agree to cooperate with the investigation. Patients with irregular distribution of skin lesions, who do not meet the characteristics of psoriasis, who refuse to cooperate, or who are not suitable to participate in this investigation for other reasons are excluded.

### 2.2. Investigation Methods

All the subjects included in the study came to the dermatology clinic of a well-known traditional Chinese medicine hospital in Jiangsu Province. According to the patient's own course of disease, each patient was initially diagnosed and an observation report was established. With the consent of the patient, a case observation form was established for the patients who met the inclusion criteria on site and archived.

### 2.3. Investigation Contents

The survey content generally includes the patient's demographic data, traditional Chinese medicine diagnosis, prescription drugs, personal distribution of skin lesions, and skin lesion morphology.

### 2.4. Body Surface Distribution Standard of Skin Lesions

Common psoriasis skin lesions are divided into head and neck (scalp, face, and neck), limbs (including upper limbs: forearm, armpit, elbow joint, hand, and nail, and lower limbs: hip, groin, thigh, knee joint, lower leg, foot, and reproductive part), body (chest, back, and abdomen), and mucous membrane.

### 2.5. Statistical Methods

All data were statistically analyzed by the combination of theoretical analysis and statistical processing of traditional Chinese medicine. Firstly, the statistical formula of mean and standard deviation rate is as follows [3]:

(1) $$\begin{array}{c} \sigma =\frac{1}{n-1}\sqrt{\overset{n}{\underset{i=1}{\sum }}{\left(x_{i}-\bar{x}\right)}^{2}},\\ \bar{x}=\frac{1}{n}\overset{n}{\underset{i=1}{\sum }}x_{i}, \end{array}$$

where *σ* is the standard deviation rate of input sequence *x*; *x*_*i*_ is the *i*th input item in the input sequence *x*; *μ* is the arithmetic mean of the input sequence *x*; *n* is the number of statistical samples.

RETRACTED

The *T* value and *P* value of bivariate *t*-check come from the bivariate *t*-check process, where *t* value is the value of the output result. When *t* > 10.000, it is considered that there is statistical consistency between the two columns of data, and the greater the *T* value, the greater the consistency; *P* value is the log value of the output result. When *P* < 0.05, it is considered that the result data is within the confidence space. When *P* < 0.01, it is considered that the result data has significant statistical significance. The smaller the *P* value, the higher the degree of confidence. Subject to the length, only the calculation algorithm of *T* value (value) is explained here, such as

(2) $$\begin{array}{c} t=\frac{\bar{X_{1}}-\bar{X_{2}}}{\sqrt{\left(\left(\left(n_{1}-1\right)\sigma_{1}^{2}+\left(n_{2}-1\right)\sigma_{2}^{2}\right)/\left(n_{1}+n_{2}-2\right)\right)\left(\left(1/n_{1}\right)+\left(1/n_{2}\right)\right)}}, \end{array}$$

where $\bar{x}$ is the arithmetic mean of the investigated sample sequence; *μ* is the average value of the reference sample sequence; *n* is the number of nodes of the investigated sample sequence; *m* is the number of nodes in the reference sample sequence; *σ*_*x* _ is the standard deviation rate of the investigated sample sequence.

The *R*^2^ value is obtained by the linear regression method under SPSS, and the *T* value and *P* value are obtained by bivariate *t*-check.

The statistical method of the *R*^2^ value is the ratio of regression residual to mean residual, as shown in

(3) $$\begin{array}{c} R^{2}=\frac{\sum {\left(\overset{\wedge }{x}-\bar{x}\right)}^{2}}{\sum {\left(x-\bar{x}\right)}^{2}}, \end{array}$$

where $\bar{x\;}$ is the arithmetic mean of the investigated sample sequence; ${\tilde{x}}_{i}$ is the *i*th regression value in the sequence; *x*_*i*_ is the *i*th input value in the sequence; *n* is the number of investigation samples.

## 3. Results

### 3.1. Analysis of Psoriasis Skin Lesions

According to the types of skin lesions in different periods, 512 investigated patients showed 186 cases (36.33%), 227 cases (44.53%), and 99 cases (19.14%) in the onset stage, stable stage, and recovery stage. The morphology of skin lesions in each period is different. Now, pathology generally believes that the pathogenic mechanism of psoriasis is related to family genetics, endocrine system, autoimmune system, mental factors, and emotions. The data from the survey report show that there are more men than women in 512 patients. See Table 1 for details.

RETRACTED

In Table 1, in the onset of psoriasis vulgaris, there are many drop-like lesions, followed by coin-like, map-like, banded, annular, shell-like, and mixed. In the stable period, most of them are drop-like, and other forms are similar. Most of the skin lesions in the recovery period are drip, coin, map, and strip. It can be seen that the skin lesions in different periods are mostly drip, coin, and map.

In order to more intuitively reflect the shape and distribution of skin lesions in different stages, visualize the data in the table to get Figure 2.

In Figure 2, it can be seen from the figure that although the patient's skin lesions will be reduced due to the improvement of his condition, most of the skin lesions are drip, coin, map, and ribbon, which is also the typical skin lesions of psoriasis vulgaris and can be regarded as the basis for the diagnosis of pathology.

### 3.2. Correlation Analysis between Psoriasis Lesions and Disease Course

With the increase of the course of disease, the condition intervention is different, and the shape of skin lesions is different. In addition, psoriasis is an easily occurring epidemic disease. Delayed post disease intervention or the disease is in the onset stage having a great impact on the morphology of skin lesions. This study conducted a bivariate *t*-test based on the course of the patient to demonstrate its correlation. See Table 2 for details:

In Table 2, the bivariate *t*-test *P* < 0.01 shows that there is a correlation between the course of disease and the form. According to the different course of disease, most of the forms of body skin lesions are common drop-like, coin-like, and map-like skin lesions at first. With the extension of the course of disease, there are more forms of body epithelial lesions. At the beginning of the disease, skin lesions may occur in common drop-like, coin-like, and map-like skin lesions. Later, due to repeated attacks, untimely intervention, improper treatment, and other reasons, the morphology of skin lesions increases, resulting in rare shell-like and mixed skin lesions.

In order to more intuitively reflect the correlation between lesion morphology and course of disease, visualize the data in the table to get Figure 3.

In Figure 3, it can be seen in the figure that the form of skin lesions increases with the increase of the course of disease. Due to the condition of psoriasis, there is no specific drug to cure the current medical level, resulting in repeated attacks of the condition, and the form of skin lesions can not be controlled. With the extension of the course of disease, the form of skin lesions on the body tends to be diversified.

RETRACTED

### 3.3. Distribution of Skin Lesions

According to the survey data statistics, the parts with higher distribution frequency of skin lesions in patients with psoriasis are lower leg (475 cases), back (441 cases), abdomen (432 cases), thigh (305 cases), forearm (286 cases), elbow (245 cases), chest (198 cases), scalp (148 cases), upper arm (132 cases), and hip (128 cases), and less distribution is mucosa (3 cases).

In Table 3, the skin lesions of 512 patients occurred most in the small leg, followed by the back, abdomen, thigh, forearm, etc., which were evenly distributed, and most of the extended side parts indicate that the extended side part had a large contact surface with the outside world, and there were relatively many opportunities for friction to be stimulated. According to the relevant reports of doctors, psoriasis may be aggravated or induced by external factors, so as to cause the repeated attack of psoriasis. In addition, the incidence of chest, scalp, and upper arm is also relatively high, and there have been similar arguments on why these parts are caused by relevant medical data, which may be related to the vascular density in them. Some substances that induce psoriasis in the dense blood vessels are easy to accumulate here, resulting in the outbreak of psoriasis induced by bacteria. Moreover, the scalp is composed of skin, fascia, and aponeurosis. Its skin is thick and dense, rich in sebaceous glands, sweat glands, hair follicles, and blood vessels. Once infected, it is not easy to spread. Therefore, the incidence of scalp is relatively high, and many chemical shampoos also increase the risk of psoriasis on the scalp.

In order to more intuitively reflect the distribution of skin lesions on the human trunk, visualize the data in the table to get Figure 4.

In Figure 4, because the pathogenesis of psoriasis is not clear, the current research believes that its etiology is mainly related to genetics, autoimmune system, endocrine system, mental factors, emotion, and other factors. The microecological imbalance of skin and mucosa will induce immune response. Now, relevant medical data demonstrate that fungal infection is related to psoriasis infection. The more skin contact areas, the more fungi stored, the higher the risk of infection. At the same time, the intersection of joints and blood vessels is easy to cause bacterial deposition and form factors inducing silver filings. Nail, face, neck, mucosa, and other blood vessels and places with less contact area, the probability of infection is relatively small.

## 4. Discussion

The 512 patients with psoriasis vulgaris in different degrees included in the study had a large age span, ranging from children to the elderly, with different onset periods and different course of disease. According to the survey data, we can know that the age of psoriasis patients is not related to the age of the patients. The youngest group is 2 years old, the largest age is 81 years old. Men are high in women. Temporary medicine has not yet clearly demonstrated the mechanism of male incidence rate higher than that of women. The general conclusion is that the bad habits of men lead to the decrease of immunity and the invasion of disease.

RETRACTED

It can be seen from Table 1 that the skin lesions of patients with psoriasis vulgaris are more common in drop shape, coin shape, and map shape and have a high frequency in the onset stage, stable stage, and recovery stage. It can be inferred that these forms are the basic skin lesions of psoriasis vulgaris. After the disease is stable in the later stage, the fusion morphology of skin lesions will also change, but ring and band are rarely seen. In the recovery period, because the number of lesions becomes less, the shape and size will shrink, and the shape and color spots will subside accordingly.

According to Bin [4], due to the unknown pathogenesis of psoriasis, targeted treatment is impossible. Most of the existing treatment methods use immune treatment. In this paper, the detection of squamous epithelial cells in recent years found that patients with skin injury diseases also have tumor risk. Contact the context, the semantic expression content has been modified to ensure that the expression meaning is complete and clear. Psoriasis Area and Severity Index (PASI) and body surface area before treatment for patients with psoriasis BSA were exponentially correlated with serum level of squamous cell carcinoma antigen (SCCA). At the same time, serum can be used as an effective index to evaluate the therapeutic effect of psoriasis and the degree of skin lesion involvement. Zhou et al. [5] have a long history of treating psoriasis with traditional Chinese medicine. They have established an independent system for this kind of disease early. They look at skin diseases from the perspective of traditional Chinese medicine, mostly from the inside, so as to deal with the problem of appearance. In this paper, psoriasis is classified as “psoriasis,” “stubborn ringworm,” and “leukoplakia.” At present, Chinese doctors mostly treat this kind of problem from blood [6]. This study starts with phlegm dampness, discusses the pathogenesis and treatment scheme of psoriasis, and puts forward new research ideas for the clinical treatment of psoriasis.

RETRACTED

It can be seen from Table 2 that there is a certain correlation between the morphology of psoriasis lesions and the course of psoriasis. Because the pathogenesis of psoriasis is unknown and repetitive, the longer the course of psoriasis, the more skin lesions distributed on the body surface and stubborn [7]. There are relevant data reports on the distribution location. Because the skin can induce psoriasis due to friction stimulation, there are more places with large body contact area. The intersection of joints and blood vessels is easy to cause bacterial deposition, which is also a factor for the formation of psoriasis [8]. In addition, there are fewer blood vessels and contact areas such as nails, face, neck, and mucous membrane. The probability of infection is relatively small.

It can be more intuitively expressed from Figure 4 that where the contact area of the body surface is large, there are more skin lesions, and most of them are symmetrically distributed, and the extended side is more than the curved side, because the extended side of the body has more opportunities to contact other objects and be stimulated by friction than the curved side. It can be inferred that the induction and exacerbation of psoriasis are related to external factors and local stimuli, because they want to cause the isomorphic reaction of psoriasis and aggravate the development of psoriasis.

## 5. Results

Psoriasis is a chronic systemic disease in China. The incidence rate of patients is about 1/1000. That is to say, one hundred of one thousand and two hundred people suffer from this disease [9]. The prevalence rate is also increasing. This disease is stubborn and recurrent, is accompanied by itching and ulceration, and has serious impact on life and personal image. It is not only physically painful but also mentally depressing. It has an adverse impact on the recovery of the disease. By studying the distribution of psoriasis lesions and the correlation between lesions, gender, and course of disease, we can improve the dialectical treatment of psoriasis, which has reference significance, and provide a new thinking direction for the treatment system theory of psoriasis [10].

There are many causes of psoriasis, and the course of disease is long and easy to relapse. The clinical treatment effect is mainly to alleviate symptoms, which can not achieve the curative effect. Moreover, there are relatively few studies on the morphology and distribution of psoriasis vulgaris, which can not be connected with its pathogenesis. Although the development of bioscience has further improved the therapeutic effect of psoriasis, it is still unable to achieve radical cure, and it is easy to relapse after drug withdrawal. It is hoped that the development of medicine in the future can solve this problem.

RETRACTED

## Figures and Tables

**Figure 1:** Age distribution of patients with psoriasis at different stages.

**Figure 2:** Morphological distribution of psoriasis vulgaris at different stages.

**Figure 3:** Visual diagram of correlation between lesion morphology and course of psoriasis vulgaris.

**Figure 4:** Distribution of psoriasis vulgaris lesions in the human body.

**Table 1:** Statistical table of skin lesions in different periods of psoriasis vulgaris (data from survey report).

Lesion type	Onset period	Stable period	Convalescence
Drop-like	73 (39.24)	76 (33.48)	35 (35.35)
Nummular	35 (18.82)	53 (23.35)	23 (23.23)
Map shape	26 (13.98)	35 (15.42)	13 (13.13)
Banded	21 (11.29)	27 (11.89)	8 (8.08)
Annular	12 (6.45)	18 (7.93)	10 (10.10)
Shell shape	13 (6.99)	13 (5.73)	8 (8.08)
Mixed	6 (3.23)	5 (2.20)	2 (2.03)

**Table 2:** Systematic table of course and lesion morphology in patients with psoriasis vulgaris (data from survey report).

Lesion type	Course of disease		*T*	*P*
	Male	Female		
Drop-like	6.36 ± 0.52	8.25 ± 0.75	0.82	0.009
Nummular	8.23 ± 0.647	9.14 ± 0.83	0.75	0.008
Map shape	5.15 ± 0.56	7.65 ± 0.68	0.79	0.007
Banded	13.45 ± 1.23	17.85 ± 2.11	0.86	0.008
Annular	16.81 ± 1.24	19.04 ± 1.65	0.91	0.009
Shell shape	20.47 ± 1.85	22.01 ± 2.17	0.93	0.007
Mixed	17.14 ± 1.23	23.54 ± 2.58	0.92	0.008

**Table 3:** Body surface distribution of psoriasis vulgaris (data from survey report).

Number	Lesion location	Number of occurrences	Proportion (%)
1	A lower leg	475	92.77
2	Back	441	86.13
3	Abdomen	432	84.38
4	Thigh	305	59.57
5	Forearm	286	55.86
6	Elbow	245	47.85
7	Chest	198	38.67
8	Scalp	148	28.90
9	Upper arm	132	25.78
10	Hips	128	25
11	Hand	107	20.9
12	Knee	74	14.45
13	Armpit	59	11.52
14	Foot	39	7.62
15	Ventral sulcus	27	5.27
16	Nail	24	4.88
17	Face	17	3.32
18	Neck	11	2.48
19	Reproduction organs	6	1.17
20	Mucous membrane	2	0.40

## Data Availability

The data underlying the results presented in the study are available within the manuscript.
